This article has been retracted.

# Dysferlin Interacts with Histone Deacetylase 6 and Increases alpha-Tubulin Acetylation

**DOI:** 10.1371/journal.pone.0028563

**Published:** 2011-12-08

**Authors:** Sabrina Di Fulvio, Bilal A. Azakir, Christian Therrien, Michael Sinnreich

**Affiliations:** 1 Neuromuscular Research Group, Departments of Neurology and Biomedicine, University, Hospital, Basel, Switzerland; 2 Neuromuscular Research Group, Montreal Neurological Institute and Hospital, McGill University, Montreal, Canada; International Centre for Genetic Engineering and Biotechnology, Italy

## Abstract

Dysferlin is a multi-C2 domain transmembrane protein involved in a plethora of cellular functions, most notably in skeletal muscle membrane repair, but also in myogenesis, cellular adhesion and intercellular calcium signaling. We previously showed that dysferlin interacts with alpha-tubulin and microtubules in muscle cells. Microtubules are heavily reorganized during myogenesis to sustain growth and elongation of the nascent muscle fiber. Microtubule function is regulated by post-translational modifications, such as acetylation of its alpha-tubulin subunit, which is modulated by the histone deacetylase 6 (HDAC6) enzyme. In this study, we identified HDAC6 as a novel dysferlin-binding partner. Dysferlin prevents HDAC6 from deacetylating alpha-tubulin by physically binding to both the enzyme, via its C2D domain, and to the substrate, alpha-tubulin, via its C2A and C2B domains. We further show that dysferlin expression promotes alpha-tubulin acetylation, as well as increased microtubule resistance to, and recovery from, Nocodazole- and cold-induced depolymerization. By selectively inhibiting HDAC6 using Tubastatin A, we demonstrate that myotube formation was impaired when alpha-tubulin was hyperacetylated early in the myogenic process; however, myotube elongation occurred when alpha-tubulin was hyperacetylated in myotubes. This study suggests a novel role for dysferlin in myogenesis and identifies HDAC6 as a novel dysferlin-interacting protein.

## Introduction

Recessive mutations in the DYSF gene cause Limb girdle muscular dystrophy type 2B (LGMD2B) [1], Miyoshi Myopathy [1] and Distal anterior compartment myopathy [2]. Dysferlin is a large type II transmembrane protein composed of two DysF domains and seven C2 domains that mediate lipid [3], [4] and protein binding interactions [5], [6], [7], [8], [9]. Dysferlin is predominantly expressed in skeletal and cardiac muscle [10], and its expression is upregulated during myogenesis [11], [12]. The subcellular localization of dysferlin is at the sarcolemma, T-tubule membranes and in intracellular vesicular compartments of as yet unknown origin [13], [14]. Dysferlin is a critical component of the calcium-dependent sarcolemmal repair complex, but recent studies have proposed additional roles for dysferlin in myogenesis [15], [16], [17], intercellular calcium signaling [18] and cellular adhesion [19]. Our recent work identified alpha-tubulin and microtubules as novel binding partners of dysferlin [6], suggesting a possible role for dysferlin in microtubule dynamics or stability.

The upregulation of microtubule acetylation is essential for myogenesis [20]. Microtubule acetylation is regulated by alpha-tubulin acetyltransferases and deacetylases, the most notable one being histone deacetylase 6 (HDAC6) [21]. Unlike most classical HDACs which are located in the nucleus and deacetylate nuclear substrates such as histones, HDAC6 contains a nuclear exclusion signal and a cytoplasmic retention signal making it a cytoplasmic enzyme [21], [22]. HDAC6 has two catalytic hdac domains used to deacetylate alpha-tubulin [21], [23], [24], cortactin [23], [25], [26] and Hsp90 [27]. HDAC6-mediated microtubule deacetylation plays important regulatory roles in microtubule dynamics [28], [29], cellular motility [23], [26], [30], [31] and motor protein motility [32].

In this study, we identified HDAC6 as a novel dysferlin interacting protein. Our results revealed that dysferlin binds to HDAC6 and alpha-tubulin, and prevents HDAC6 from deacetylating its substrate, alpha-tubulin. We also demonstrated that inhibition of HDAC6 activity in the early stages of myoblast differentiation results in impaired myogenesis, whereas increased microtubule acetylation in myotubes results in myotube elongation. We suggest that the increasing dysferlin expression observed during myogenesis could be required to decrease HDAC6-mediated microtubule deacetylation.

## Results

### Dysferlin interacts with HDAC6 and prevents alpha-tubulin deacetylation

We had previously performed a mass spectrometric analysis of the dysferlin protein complex [6] and identified HDAC6 as a potential dysferlin interactor. This protein was also identified in another study [33]. To confirm this interaction, we performed binding assays using recombinant and native dysferlin and HDAC6 proteins. Recombinant dysferlin was able to bind either to recombinant FLAG-HDAC6 expressed in HEK293T cells (Figure 1A) or to native HDAC6 from homogenized murine testes (Figure 1B), which are a rich source of the enzyme. Co-immunoprecipitation assays performed in mouse skeletal muscle extracts showed that native dysferlin co-immunoprecipitated with native HDAC6 (Figure 1C).

**Figure 1:** Dysferlin co-immunoprecipitates with HDAC6. (A) HEK293T cells were transfected with GFP-myc-dysferlin (GFP-myc-Dysf) and FLAG-HDAC6, and recombinant dysferlin was immunoprecipitated (IP) with anti-myc antibodies. Immunoprecipitates were separated by SDS-PAGE and immunoblotted (IB) with the indicated antibodies. SM = starting material, 5% of total protein loaded. (B) GFP-myc-dysferlin (GFP-myc-Dysf) or GFP vector were transfected in HEK293T cells, immunoprecipitated with anti-GFP antibodies and incubated with testes homogenate from wildtype C57Bl/6 mice, which is a rich source of HDAC6. Immunoprecipitates were immunoblotted with the indicated antibodies. Alpha-tubulin was used as a loading control. (Right panel) HDAC6 protein levels in testes of wildtype C57Bl/6 mice (WT) versus HDAC6 knockout mice (KO), which were immunoblotted with anti-HDAC6 antibodies to demonstrate the specificity of the detected band. (C) Native dysferlin was immunoprecipitated with anti-dysferlin antibodies in mouse skeletal muscle extracts. Immunoprecipitates were separated by SDS-PAGE and immunoblotted with anti-dysferlin and anti-HDAC6 antibodies. (D) GFP-myc-dysferlin and FLAG-HDAC6 were overexpressed in Cos7 cells. Cells were fixed and immunostained with anti-GFP and anti-FLAG antibodies. (E) 134/04 cells were transfected with FLAG-HDAC6 and differentiated into myotubes. Cells were fixed and immunostained with anti-dysferlin and anti-FLAG antibodies. Scale bar: 20 µm.

To determine if dysferlin and HDAC6 co-localized in the same subcellular compartment, GFP-myc-dysferlin and FLAG-HDAC6 were transfected into Cos7 cells. Immunostaining showed partial co-localization between the two proteins in the cytoplasm and in the vicinity of the plasma membrane (Figure 1D). To determine if the proteins co-localized in muscle cells, FLAG-HDAC6 was transfected into a human myoblast cell line (134/04), which harbours two wildtype DYSF alleles, and cells were differentiated into myotubes. Immunostaining with anti-dysferlin and anti-FLAG antibodies demonstrated that the proteins partially co-localized in the cytoplasm and in the vicinity of the plasma membrane (Figure 1E).

To identify which of dysferlin's seven C2 domains could be involved in the interaction with HDAC6, we constructed a series of single C2 domain deletion mutants from full-length wildtype (WT) dysferlin, which harbours an N-terminal GFP tag and C-terminal myc-His tags (Figure 2A). Each mutant (ΔC2A to ΔC2G), or WT dysferlin or a GFP vector was expressed in HEK293T cells, immobilized on nickel affinity beads, and incubated either with recombinant FLAG-HDAC6 (Figure 2B) or with native HDAC6 from homogenized murine testes (Figure 2C). In both assays, dysferlin's C2D domain was required for the interaction with HDAC6.

**Figure 2:** Dysferlin binds HDAC6 through its C2D domain and prevents alpha-tubulin deacetylation. (A) Schematic of dysferlin C2 domain deletion constructs. (B) Wildtype dysferlin (WT), dysferlin deletion mutants (ΔC2A through ΔC2G) or GFP vector were transfected in HEK293T cells, pulled-down on Ni-NTA beads, and incubated with FLAG-HDAC6-transfected HEK293T cell lysates. Immunoprecipitates were immunoblotted with the indicated antibodies. (Right panel) FLAG-HDAC6 expression levels in transfected HEK293T cell lysates, immunoblotted with anti-FLAG antibody. (C) Wildtype dysferlin (WT), dysferlin deletion mutants (ΔC2A through ΔC2G) or GFP vector were transfected in HEK293T cells, pulled-down on Ni-NTA beads, and incubated with murine testes homogenate. Immunoprecipitates were immunoblotted with the indicated antibodies. (Right panel) This western blot is identical to the one displayed in Fig. 1B. (D) Cell lysates from (C) were immunoblotted for alpha-tubulin acetylation levels. Similar results observed with cell lysates from (B) (not shown).

Given that HDAC6 is a major alpha-tubulin deacetylase, we assayed for dysferlin's effect on alpha-tubulin acetylation. Alpha-tubulin acetylation levels increased in HEK293T cells expressing wildtype dysferlin (WT) or the following C2 domain deletion mutants: ΔC2B, ΔC2C, ΔC2E, ΔC2F and ΔC2G (Figure 2D). Cells expressing ΔC2A or ΔC2D showed no change in alpha-tubulin acetylation levels compared to GFP vector-expressing cells, indicating that dysferlin requires its C2A and C2D domains to prevent HDAC6 from deacetylating alpha-tubulin.

### Dysferlin requires alpha-tubulin binding to prevent HDAC6 from deacetylating alpha-tubulin

We recently showed that dysferlin interacts with alpha-tubulin through its C2A and C2B domains, although this interaction is weaker with the C2B domain than with the C2A domain [6]. Figures 2B and 2C show that the ΔC2A deletion mutant interacted less strongly with alpha-tubulin when compared to wildtype dysferlin or the other six deletion mutants, which is in agreement with our previously published results. Notably, the interaction was not fully abolished since the ΔC2A deletion mutant retains its C2B domain, which also interacts with alpha-tubulin, albeit weakly. Theorizing that dysferlin requires both of its alpha-tubulin binding domains to interact with HDAC6, we used a truncated dysferlin mutant lacking its three N-terminal C2 domains, but retaining its DysF domains (DD) and the transmembrane domain (TM) (DD-DEFG-TM) (Figure 3A). As expected, this N-terminally truncated mutant did not pull down alpha-tubulin, and also showed weaker binding to HDAC6 (Figure 3B). This suggests that dysferlin also requires both of its alpha-tubulin binding domains (C2A and C2B) to fully interact with HDAC6.

**Figure 3:** Dysferlin requires its alpha-tubulin binding domains to bind HDAC6 and prevent alpha-tubulin deacetylation. (A) Schematic of dysferlin truncation construct (DD-DEFG-TM). (B) Wildtype dysferlin (WT), dysferlin deletion mutants ΔC2A and ΔC2D, or DD-DEFG-TM were transfected in HEK293T cells, pulled-down on Ni-NTA beads, incubated with murine testes homogenate and immunoblotted with the indicated antibodies. (C) Cell lysates from (B) were immunoblotted for alpha-tubulin acetylation levels. (D) FLAG-HDAC6 was co-transfected with wildtype dysferlin (WT), dysferlin deletion mutants (ΔC2A and ΔC2D), dysferlin truncation (DD-DEFG-TM) or GFP vector in HEK293T cells, immunoprecipitated with anti-alpha-tubulin antibodies, and immunoblotted with the indicated antibodies. As controls, cell lysates were immunoprecipitated without antibodies (CTL) or with anti-IgG antibodies (IgG).

We assessed whether the truncated mutant DD-DEFG-TM could affect alpha-tubulin acetylation levels in HEK293T cells. As shown in Figure 3C, DD-DEFG-TM did not alter the amount of acetylated alpha-tubulin, similarly to ΔC2A and ΔC2D deletion mutants. In agreement with Figure 2D, these results highlight the importance of dysferlin's C2A domain in preventing alpha-tubulin deacetylation.

Having shown that dysferlin's alpha-tubulin binding domains are important for impairing HDAC6-mediated deacetylation of alpha-tubulin, we theorized that dysferlin may be having this effect by affecting HDAC6's ability to interact with its substrate. To assess how dysferlin may affect HDAC6's interaction with alpha-tubulin, we performed an alpha-tubulin immunoprecipitation assay in HEK293T cells expressing FLAG-HDAC6 along with either wildtype dysferlin (WT), the ΔC2A or ΔC2D deletion mutants, or with the truncated mutant (DD-DEFG-TM). As shown in Figure 3D, in the absence of dysferlin, HDAC6 is able to bind to alpha-tubulin. However, in the presence of full-length dysferlin, alpha-tubulin no longer pulled down HDAC6, but only dysferlin. This effect was only observed if dysferlin retained its C2D domain as well as its alpha-tubulin binding C2A and C2B domains; if these domains were deleted, dysferlin did not prevent HDAC6 from interacting with alpha-tubulin. This is demonstrated by the ΔC2D and DD-DEFG-TM constructs, which showed an unimpaired HDAC6 interaction with alpha-tubulin (Figure 3D). Because the ΔC2A construct still had partial alpha-tubulin binding capabilities and an intact C2D domain, it was able to decrease HDAC6's interaction with alpha-tubulin, but not abolish it completely as did wildtype dysferlin. These results suggest that dysferlin prevents HDAC6 from interacting with its substrate, thus hindering alpha-tubulin deacetylation.

### Dysferlin expression increases alpha-tubulin acetylation and resistance to microtubule depolymerization

Having demonstrated that recombinant dysferlin affects alpha-tubulin acetylation levels in HEK293T cells, we assessed whether native dysferlin expression also affected alpha-tubulin acetylation in muscle cells. We used three human myoblast cell lines: 134/04 cells harbouring two wildtype DYSF alleles, ULM1/01 cells harbouring two nonsense DYSF alleles, and 180/06 cells harbouring one missense DYSF allele and one nonsense DYSF allele. The cells were cultured, lysed and immunoblotted for acetylated-alpha-tubulin and alpha-tubulin levels. As shown in Figure 4A, wildtype cells (134/04) had higher levels of acetylated alpha-tubulin than dysferlin-deficient cells (180/06 and ULM1/01). To confirm that the effect was specific to dysferlin expression, wildtype dysferlin (WT) or the ΔC2A deletion mutant was overexpressed in 134/04 cells. In agreement with Figures 2D and 3C, dysferlin overexpression in muscle cells resulted in increased alpha-tubulin acetylation levels, whereas expression of the ΔC2A deletion mutant did not affect alpha-tubulin acetylation (Figure 4B).

**Figure 4:** Dysferlin expression increases alpha-tubulin acetylation in muscle cells. (A) 134/04, 180/06 and ULM1/01 cell lysates were immunoblotted with anti-dysferlin and anti-acetylated alpha-tubulin antibodies. Alpha-tubulin was used as a loading control. (B) GFP-dysferlin wildtype (WT) or GFP-dysferlinΔC2A (ΔC2A) were transfected into 134/04 myoblasts. Transfected and untransfected (CTL) cell lysates were separated by SDS-PAGE and immunoblotted with the indicated antibodies.

Microtubule post-translational modifications occur subsequent to microtubule stabilization; therefore alpha-tubulin acetylation can be considered as a marker of stabilized microtubules [34]. Stabilized microtubules are more resistant to microtubule depolymerization. We theorized that the increased alpha-tubulin acetylation levels observed in dysferlin-expressing cells were indicative of a pool of microtubules with increased resistance to depolymerization. To test this theory, we employed cold-induced and Nocodazole-induced microtubule depolymerization assays. In the cold-induced depolymerization assay, 134/04, 180/06 and ULM1/01 cells were incubated at 4°C for increasing lengths of time, and microtubule resistance was assessed by the amount of acetylated alpha-tubulin remaining post-treatment. As shown in Figures 5A and 5E, 134/04 cells retained significantly higher acetylated alpha-tubulin levels following cold treatments (30, 45 and 60 min) than dysferlin-deficient 180/06 and ULM1/01 cells. In the Nocodazole-induced depolymerization assay, 134/04, 180/06 and ULM1/01 cells were treated with increasing concentrations of Nocodazole, and microtubule resistance to depolymerization was assessed by the amount of acetylated alpha-tubulin remaining post-treatment. As shown in Figures 5B and 5F, 134/04 cells retained significantly higher acetylated alpha-tubulin levels following Nocodazole treatment (3 µg/ml and 9 µg/ml) than dysferlin-deficient 180/06 and ULM1/01 cells. To demonstrate that the effect was specific to dysferlin expression, wildtype dysferlin (WT) or ΔC2A were expressed in HEK293T cells, which were similarly treated with Nocodazole. As shown in Figures 5C and 5G, cells transfected with WT dysferlin showed significantly more acetylated alpha-tubulin levels post-Nocodazole treatment when compared to untransfected (CTL) cells. In agreement with our previous results, this effect required dysferlin's C2A domain, as cells transfected with ΔC2A showed acetylated alpha-tubulin levels that were comparable to untransfected (CTL) cells. These results suggest that dysferlin expression correlates with increased microtubule resistance to Nocodazole treatment, indicative of the presence of a larger pool of stable microtubules.

**Figure 5:** Dysferlin expression increases resistance to microtubule depolymerization. (A) 134/04, 180/06 and ULM1/01 cells were incubated at 4°C for increasing lengths of time. Cell lysates were immunoblotted with the indicated antibodies. To equalize the baseline (0 min) acetylated alpha-tubulin levels in the 180/06 and ULM1/01 cells with those of the 134/04 cells, the intensity of the bands was linearly increased post-acquisition. (B) 134/04, 180/06 and ULM1/01 cells were untreated (Unt), mock-treated (Mock) or treated with increasing concentrations of Nocodazole. Cell lysates were immunoblotted with the indicated antibodies. To equalize the baseline (Unt) acetylated alpha-tubulin levels in the 180/06 and ULM1/01 cells with those of the 134/04 cells, the intensity of the bands was linearly increased post-acquisition. (C) GFP-dysferlin wildtype (GFP-Dysf WT) or GFP-dysferlinΔC2A (GFP-DysfΔC2A) were transfected into HEK293T cells. Transfected and untransfected (CTL) cells were treated with increasing concentrations of Nocodazole. Cell lysates were immunoblotted with the indicated antibodies. (D) 134/04, 180/06 and ULM1/01 cells were untreated (Unt) or treated with 2.5 µg/ml Nocodazole, then the drug-containing media was replaced with fresh media and cells were allowed to recover for the indicated lengths of time. Cell lysates were immunoblotted with the indicated antibodies. To equalize the baseline (Unt) acetylated alpha-tubulin levels in the 180/06 and ULM1/01 cells with those of the 134/04 cells, the intensity of the bands was linearly increased post-acquisition. (E, F, G) The ratio of acetylated alpha-tubulin∶alpha-tubulin at each time point or Nocodazole concentration was normalized to 134/04 levels to equalize starting values. * indicates that 134/04 values or GFP-Dysf WT values were significantly greater (p<0.05) than 180/06 and ULM1/01 levels (E, F) or CTL and ΔC2A levels (G), at the indicated time point or concentration. (H) The ratio of acetylated alpha-tubulin: alpha-tubulin was calculated for each time point and normalized to 134/04 levels to equalize starting values. *, # and+indicate that the value at the indicated time point is significantly different (p<0.05) than the Unt value for 134/04, 180/06, ULM1/01, respectively.

Once the microtubule depolymerising agent is removed, microtubules will repolymerize during a recovery phase [35]. To study the effect of dysferlin expression on microtubule recovery from Nocodazole treatment, cells were treated with Nocodazole for 45 min and then the drug-containing media was removed and replaced with fresh media, thus allowing repolymerization of microtubules. After defined lengths of time, the alpha-tubulin acetylation levels were measured as a marker of microtubule repolymerization and stabilization. Figures 5D and 5H show that dysferlin expression (134/04 cells) resulted in faster recovery from Nocodazole treatment than was observed in dysferlin-deficient cells (180/06 or ULM1/01 cells). Taken together, these results show that dysferlin expression increases cellular alpha-tubulin acetylation levels, as well as promotes microtubule resistance to, and recovery from, induced depolymerization.

### Hyperacetylation of alpha-tubulin impairs myogenesis

Microtubule acetylation and dysferlin expression are both upregulated during myogenesis [11], [20]. To demonstrate this in our cultured human myoblasts, 134/04 cells were cultured in differentiation media for up to four days to induce myotube formation. Lysates from these cells and from homogenized mouse skeletal muscle were immunoblotted for dysferlin and acetylated-alpha-tubulin levels. Results showed that both dysferlin and acetylated alpha-tubulin levels increased during myogenic differentiation (Figure 6A). Immunofluorescent staining for acetylated alpha-tubulin levels in 134/04 cells show significantly higher levels in differentiated myotubes than in undifferentiated myoblasts (Figure 6B). On the other hand, dysferlin-deficient myoblasts (180/06) do not differentiate into myotubes and the acetylated alpha-tubulin were unchanged even after four days in differentiation media (Figure 6B).

**Figure 6:** Dysferlin and acetylated alpha-tubulin levels increase during differentiation. (A) 134/04 cells were cultured in differentiation media for the indicated number of days. Cell lysates from these cells and mouse skeletal muscle extract were immunoblotted with the indicated antibodies. (B) 134/04 cells and 180/06 cells were cultured in differentiation media for 0 days or 4 days to induce myotube formation. Cells were fixed and immunostained with anti-acetylated alpha-tubulin antibodies and DAPI. Images were captured at the same fluorescence intensity and gain to compare alpha-tubulin acetylation levels between cells. Scale bar: 20 µm.

Our data suggests that upregulated dysferlin expression would increase microtubule acetylation via its interaction with HDAC6. Given that microtubule acetylation is a late-stage event in myogenesis, we theorized that early upregulation of dysferlin would result in prematurely increased acetylation levels, which could have detrimental effects on myotube formation. However, dysferlin has previously been shown to play a role in myogenesis [16], [17], for instance by affecting myogenin expression [16]. Therefore, it would not be possible to attribute any potential myogenic effect from overexpressing dysferlin in dysferlin-deficient myoblasts specifically to dysferlin's role on alpha-tubulin acetylation. Therefore, we used instead an HDAC6-specific inhibitor that causes alpha-tubulin hyperacetylation, to mimic the effect of dysferlin overexpression on alpha-tubulin acetylation specifically. Tubastatin A is a more selective derivative of the HDAC6 specific inhibitor Tubacin, which specifically inhibits alpha-tubulin deacetylation without affecting HDAC6's other substrates [24], [29], [30], [36], [37].

Myoblast differentiation assays were performed by treating 134/04 human myoblasts and C2C12 murine myoblasts continuously with Tubastatin A beginning at different stages of myoblast differentiation: at the stage when myoblasts were undifferentiated (Day 0), at the stage when myoblasts were beginning to form myotubes (Day 2) or at the stage when myotubes were terminally differentiated (Day 4) (Figure 7A). Acetylated alpha-tubulin levels in the cell lysates were assessed to confirm Tubastatin A efficacy (Figure 7B). The cells were immunostained for desmin and DAPI (Figure 7C). Desmin-stained myotubes were counted and categorized according to length (Figure 7D). The number of nuclei per myotube was also counted and the average number of nuclei in each category of myotube length was determined (Figure 7E).

**Figure 7:** Effect of HDAC6 inhibition on myotube formation. (A) C2C12 or 134/04 myoblasts were seeded in growth media on Day -1, then switched to differentiation media on Day 0. Cells were mock-treated (Mock) or treated with 7.5 µM Tubastatin A beginning on different days post-induction of myogenic differentiation (Day 0, Day 2, Day 4). On Day 5, cells were fixed and stained with an anti-desmin antibody and DAPI. (B) Alpha-tubulin acetylation levels were assayed to confirm Tubastatin A efficacy. (C) Representative immunofluorescence images of desmin-stained myotubes in each treatment regime. Scale bar: 60 µm. (D) Desmin-stained myotubes were categorized by their myotube length, and plotted against their relative number. (E) Desmin-stained myotubes were counted for their average number of nuclei and categorized by myotube length as in (D). * in (D) and (E) indicates p<0.05, significantly different from mock-treated myotubes in the same category. ** indicates that no myotubes were observed in the indicated category. (F) Absolute number of desmin-stained myotubes were counted and categorized by treatment regime. * indicates p<0.05, significantly different from Mock-treated. Shown here are results for C2C12 cells; similar results were obtained for 134/04 cells (not shown).

When treated early (Day 0, Day 2), myotube formation was significantly impaired (Figure 7C), resulting in fewer myotubes being formed (Figure 7F). The myotubes that did form were significantly shorter than mock-treated myotubes; additionally no long myotubes (>500 µm) were produced (Figure 7D). Conversely, when myotubes were hyperacetylated after terminal differentiation (Day 4), a significantly larger proportion of myotubes were longer than 600 µm when compared to mock-treated cells (Figure 7D), indicating that myotube length was increased. The average number of nuclei in this category of myotubes (>600 µm) was not significantly different from mock-treated cells (Figure 7E), indicating that the increased length was not due to increased myoblast fusion. These results suggest that microtubule hyperacetylation in the early-stages of myoblast differentiation is detrimental to myogenesis, whereas late-stage hyperacetylation can promote myotube elongation.

## Discussion

Dysferlin is a multi-C2 domain transmembrane protein involved in skeletal muscle membrane repair, and has also been implicated in myogenesis, cellular adhesion and intercellular calcium signaling. In light of the growing evidence supporting dysferlin's multifunctionality, understanding dysferlin's biology will depend on identifying its interacting proteins. To this end, we previously undertook a proteomic search through the analysis of immunoprecipitated proteins from mouse skeletal muscle using liquid chromatography-tandem mass spectrometry [6]. In this study, we identified HDAC6 as a novel dysferlin binding partner, and present a new function for dysferlin in the modulation of alpha-tubulin acetylation via an interaction with this microtubule deacetylase.

We show that dysferlin prevents HDAC6 from deacetylating alpha-tubulin by physically binding both to the enzyme via its C2D domain and to the substrate, alpha-tubulin, via its alpha-tubulin binding C2A and C2B domains. Consequently, dysferlin expression increased the alpha-tubulin acetylation levels in muscle cells. The increased alpha-tubulin acetylation levels in dysferlin-expressing cells reflect a larger pool of stable microtubules, which we showed are more resistant to Nocodazole-induced depolymerization and cold-induced depolymerization. Dysferlin expression also promoted faster microtubule recovery from depolymerization, resulting in more microtubules being repolymerized, stabilized and consequently post-translationally modified by acetylation.

A question that emerges from this study is how dysferlin prevents HDAC6 from interacting with its substrate. One possibility is that dysferlin targets HDAC6 via its C2D domain and then reinforces the interaction by binding to alpha-tubulin. Dysferlin may then directly or indirectly block HDAC6 from interacting with alpha-tubulin, thus inhibiting its ability to deacetylate microtubules. This is demonstrated by the observation that (i) loss of dysferlin's C2A domain resulted in a decreased interaction between HDAC6 and alpha-tubulin (Figure 3D) and (ii) loss of both of dysferlin's C2A and C2B domains resulted in decreased binding between dysferlin and HDAC6 (Figure 3B). Another possibility is that dysferlin binds to alpha-tubulin via its C2A and C2B domains, and uses its HDAC6-binding C2D domain to block or dislodge the enzyme from alpha-tubulin. This is suggested by the alpha-tubulin co-immunoprecipitation experiment (Figure 3D), in which full-length dysferlin was pulled down by alpha-tubulin but HDAC6 was not. It is further possible that dysferlin may sequester HDAC6 away from its substrate, as Figure 2 demonstrated a strong interaction between full-length dysferlin and HDAC6 that may be indicative of a cytoplasmic subpopulation of the two proteins which would not be observed in the alpha-tubulin co-immunoprecipitation experiment. Further studies would be required to elucidate the mechanism involved in dysferlin's interaction with HDAC6.

To study the effect of alpha-tubulin hyperacetylation on myogenesis, we used Tubastatin A, a selective HDAC6 inhibitor. When HDAC6 was inhibited early during differentiation, myotube formation was impaired, whereas HDAC6 inhibition in differentiated myotubes promoted myotube elongation.

Impaired myogenesis arising from early microtubule hyperacetylation could be caused by disrupted microtubule dynamics and protein targeting. Dynamic microtubules are required to target the cell periphery and HDAC6 inhibition has been shown to decrease microtubule dynamics [28], [29]. Premature HDAC6 inhibition could promote a more stabilized microtubule pool, thus impairing the microtubule reorganization from a radial configuration in undifferentiated myoblasts to the organized longitudinal array observed in differentiated myotubes. Alpha-tubulin hyperacetylation would also compromise the microtubule tracks used for protein, vesicle and organelle delivery. Proteins, such as CLASPs, depend on spatial cues along microtubules to locally regulate microtubule dynamics, which are provided by discrete regions of microtubule acetylation [38]. Such signals would be disrupted by microtubule hyperacetylation.

In myotubes, on the contrary, increased microtubule acetylation could promote myotube elongation by affecting microtubule polarization and motor protein movement. It has been proposed that the linear microtubule array in differentiated myotubes directly promotes myotube elongation by providing polarization, which restricts myotube elongation to a single axis [39], [40]. Furthermore, microtubule acetylation enhances kinesin-1 recruitment to microtubules and anterograde movement along microtubules [32], [41], thus permitting the delivery of cytoskeletal remodelling factors, target site recognition molecules or adhesion molecules [42], [43]. Additionally, microtubule acetylation has been proposed to designate stabilized microtubules extending all the way to a destination [32], thus promoting the delivery of proteins necessary for myotube formation and elongation.

Dysferlin expression is upregulated during myogenesis, with higher levels being observed in differentiated myotubes [11], [12]. We showed that Tubastatin A treatment of undifferentiated myoblasts resulted in impaired myotube formation, such as is observed in dysferlin-deficient myoblasts [16], [17]. Thus, our study suggests that early expression of dysferlin would promote premature microtubule hyperacetylation by way of inhibiting HDAC6, which would impair myotube formation. On the other hand, later expression of dysferlin would promote myotube formation and elongation through increased microtubule acetylation. This could explain the temporal expression pattern of dysferlin during myogenesis. The observed reduction in the number of long myotubes, and concomitant increase in short myotubes, in dysferlin-deficient cell cultures [15], [17] is in keeping with our explanation for the temporally-regulated dysferlin expression during myogenesis. We theorize that the impaired myotube elongation in these cells might in part be explained by active HDAC6, which would maintain low levels of acetylated microtubules.

For the design of dysferlin gene therapies, our study would caution against the use of ubiquitous promoters or promoters expressed early in muscle development, such as CMV and CAG [44]. Instead our data would support the use of promoters that are expressed at later stages of muscle differentiation, such as C5–12 [45] and the human α-skeletal actin promoter [44].

In summary, we have identified HDAC6 as a novel dysferlin-interacting protein, and demonstrated that the interaction between these two proteins is mediated by dysferlin's C2D domain and that dysferlin prevents HDAC6 from deacetylating alpha-tubulin by physically binding to both the enzyme and to the substrate, alpha-tubulin. Finally, we demonstrated the importance of late alpha-tubulin hyperacetylation during the myogenic process, and propose that dysferlin may act as an inhibitor of HDAC6-mediated microtubule deacetylation during myogenesis.

## Materials and Methods

### Ethics Statement

All animals were handled in strict accordance with good animal practice as defined by the relevant national and/or local animal welfare bodies, and all animal work was approved by the appropriate committee: Cantonal Veterinary Office of Basel, Switzerland (Approval IDs: 2391 and 51). Primary human myoblasts (134/04, 180/06 and ULM1/01) were obtained from EuroBioBank (www.eurobiobank.org) along with the required regulatory permissions (Approval ID: LMU 107/01).

### Cell Cultures

C2C12 murine myoblasts and Human embryonic kidney derived cells (HEK293T) were purchased from ATCC (Burlington, Ontario) (ATCC number CRL-1573 and CRL-1772 respectively) [6]. 134/04 cells contain two wildtype DYSF alleles; 180/06 cells harbour one DYSF allele containing the missense mutation C1663T (Arg555Trp) and an additional null allele 3708delA (D1237TfsX24). Myoblast culture ULM1/01 harbours two null alleles: a C4819T (R1607X) substitution and a 5085delT (F1695LfsX48) deletion. Myoblast cultures were immortalized with a retrovirus carrying the E6E7 early region from human papillomavirus type 16, as previously described [46]. Cells were maintained in growth media (10% FBS (Gibco) in DMEM (Sigma)).

### Plasmids, Constructs, Antibodies

FLAG-tagged HDAC6 was purchased from AddGene (Plasmid number 13823). The GFP-myc-His-Dysferlin was a kind gift from Dr. K. Bushby, Newcastle [6], [47]. GFP-tagged dysferlin C2-domain deletion mutants were cloned from the full-length dysferlin construct, each having a single C2 domain deleted. Deletion of the C2 domains coding region was performed by PCR mutagenesis using domain spanning oligonucleotides and the QuikChange Site-Directed Mutagenesis Kit (Stratagene), using either the single [48] or double mutagenic primers approach (Supplementary Table S1). The procedure was performed according to the manufacturer's protocols. Dysferlin truncation construct (DD-DEFG-TM), retaining its DysF domains (DD) and C2D-E-F-G domains (DEFG) and transmembrane domain (TM), was cloned from the full-length dysferlin construct. The C-terminal DD-DEFG-TM portion was first cloned into the pcDNA/TO/myc-His vector (Invitrogen), and then eGFP was added N-terminally in a second cloning step (Supplementary Table S1). All clones were sequenced in both DNA strands to confirm the deletions and the conservation of the reading frame.

Mouse monoclonal antibodies against dysferlin, FLAG and acetylated alpha-tubulin were purchased from Vector Laboratories, Sigma and Santa Cruz, respectively. Rabbit polyclonal antibodies against HDAC6 and alpha-tubulin were purchased from Abcam. Rabbit polyclonal GFP antibody was purchased from Invitrogen. Secondary antibodies, Alexa Fluor 680 goat anti-mouse IgG and InfraRed Dye 800 goat anti-rabbit IgG, were purchased from Invitrogen and Rockland, respectively.

### Co-immunoprecipitation assays, pulldown assays and Western blot

Cells were transfected using Lipofectamine 2000 (Invitrogen) in OptiMEM (Gibco) for 48 hours. Cells were lysed and immunoprecipitated (IP) as previously described [6]. For pulldown assays, dysferlin-transfected cells were similarly lysed, and supernatants were incubated with His-Select Nickel Affinity (Ni-NTA) Gel (Sigma) in the presence of 20 mM Imidazole (Sigma) overnight at 4°C, washed with 50 mM Imidazole, and incubated with FLAG-HDAC6-expressing cell extracts (similarly prepared), or with wildtype murine testes homogenates (prepared as described [6]), overnight at 4°C in IP buffer. Beads were washed with 50 mM Imidazole and separated by SDS-PAGE. Proteins were transferred onto PVDF membranes, blocked in Blocking buffer (3% Top-Block (LubioScience) with 0.05% sodium azide (Sigma)), incubated overnight with the indicated antibodies in Blocking buffer plus 0.05% Tween-20 (Merck) and detected by Fluorimetric analysis (Odyssey version 2.1.12). All experiments were performed in triplicates. Densiometric analysis was performed using ImageJ 1.43 u (NIH, USA). Statistical analysis was performed using the Student's T-test with a significance level of at least 0.05.

### Microtubule depolymerization and recovery assays

For microtubule depolymerization assays, cells were grown to confluency and treated for 45 min with the indicated concentration of Nocodazole (Sigma) in growth media, or alternatively incubated at 4°C for the indicated lengths of time. Cells were washed, lysed and western blotted as described above. For recovery experiments, cells were treated similarly, then Nocodazole was replaced with fresh media and cells were incubated at 37°C, 5% CO_2_ for the indicated lengths of time. Cells were washed, lysed and western blotted as described above. All experiments were performed in triplicates. Densiometric analysis was performed using ImageJ 1.43 u (NIH, USA). Statistical analysis was performed using the Student's T-test with a significance level of at least 0.05.

### Immunofluorescence assays

Cells were grown on matrigel-coated coverslips in growth media or in differentiation media for four days to induce myotube formation. Cells were fixed with 4% paraformadehyde (PFA) for 20 min, blocked 15 min in 2% fish skin gelatin, 1% normal goat serum, 0.15% Triton X-100 in PBS and incubated for 1 hour at room temperature with the indicated antibodies. Incubation with anti-FLAG antibodies was performed at 37°C for 2 hours. Cells were captured on a LSM 710 inverted confocal microscope (Zeiss) and analyzed using Zen 2009 LE software (Zeiss). All experiments were performed in triplicates.

### Myoblast differentiation assays

Cells were grown to 80% confluency then switched to differentiation media (2% horse serum (Sigma) in DMEM). Cells were treated with 7.5 uM Tubastatin A (BioVision, LubioScience) either at the same time at media switch (Day 0 or D0), after 48 hours in differentiation media (Day 2 or D2) or after 72 hours (Day 4 or D4). 24 hours later (Day 5), cells were lysed and western blotted as described above, or fixed with 4% PFA for 20 min, blocked 15 min in 2% fish skin gelatin, 1% normal goat serum, 0.15% Triton X-100 in PBS, then stained for desmin and DAPI. Myotubes were imaged with a Leica DMI6000B fluorescence microscope with the Volocity 5.2.0 software (Improvision Ltd) and analyzed with AnalySIS^D^ 5.0 (Soft-imaging). All experiments were performed in triplicates. Statistical analysis was performed using the Student's T-test with a significance level of at least 0.05.

## Supporting Information

Table S1 **Primers used for dysferlin C2 domain deletion constructs.** List of primers used to clone dysferlin C2 deletion constructs from full-length dysferlin. Residues that were deleted from each construct are indicated. Deletion of the C2 domains coding region was performed by PCR mutagenesis using either the single or double mutagenic primers approach (see Materials and Methods).
(DOC)
